# Multiscale U-Net with Spatial Positional Attention for Retinal Vessel Segmentation

**DOI:** 10.1155/2022/5188362

**Published:** 2022-01-10

**Authors:** Congjun Liu, Penghui Gu, Zhiyong Xiao

**Affiliations:** ^1^School of Computer Science, Jiangsu University of Science and Technology, Zhenjiang 212100, China; ^2^School of Artificial Intelligence and Computer Science, Jiangnan University, Wuxi 214122, China

## Abstract

Retinal vessel segmentation is essential for the detection and diagnosis of eye diseases. However, it is difficult to accurately identify the vessel boundary due to the large variations of scale in the retinal vessels and the low contrast between the vessel and the background. Deep learning has a good effect on retinal vessel segmentation since it can capture representative and distinguishing features for retinal vessels. An improved U-Net algorithm for retinal vessel segmentation is proposed in this paper. To better identify vessel boundaries, the traditional convolutional operation CNN is replaced by a global convolutional network and boundary refinement in the coding part. To better divide the blood vessel and background, the improved position attention module and channel attention module are introduced in the jumping connection part. Multiscale input and multiscale dense feature pyramid cascade modules are used to better obtain feature information. In the decoding part, convolutional long and short memory networks and deep dilated convolution are used to extract features. In public datasets, DRIVE and CHASE_DB1, the accuracy reached 96.99% and 97.51%. The average performance of the proposed algorithm is better than that of existing algorithms.

## 1. Introduction

Many eye-related diseases can lead to structural characteristics changes of the retinal vessel in fundus images. Therefore, fundus retinal vessel segmentation plays a significant role in the detection and diagnosis of these eye diseases, such as diabetic retinopathy, hypertension, and arteriosclerosis [1]. However, the manually visual vessel segmentation method requires professional doctors to label blood vessels manually, which not only is time-consuming but also can be easily affected by subjective factors. Therefore, in recent years, a variety of methods have been proposed for retinal vessel segmentation tasks, including unsupervised methods and supervised methods [2].

Unsupervised learning methods do no't use any annotation as a reference and aim to extract blood vessels based on one or more characteristics of the blood vessel. For example, Xiao et al. [3] used an improved level set method to minimize the proposed energy function to identify blood vessels in retinal images. Azzopardi et al. [4] designed the B-COSFIRE filter, which can accurately detect the trunk and end of blood vessels in different directions. Unsupervised algorithms do no't need to rely on annotated vascular images, but they are less robust and have no learning ability. In recent years, with the development of deep neural networks, good results have been achieved in the field of medical image processing [5–7]. Therefore, more and more algorithms based on deep learning are used for retinal vessel segmentation.

Existing deep learning-based retinal vessel segmentation models can be classified into four groups according to network structure [8]. The first group is to use only a few layers of CNN to segment blood vessels. These models can only segment the basic structure of vessels and canno't segment the boundary and thin vessels. For example, The CNN model with multiple convolutional layers was proposed by Uysal et al. [9]. The proposed model can do pixel-level recognition but canno't detect vessels very well. The second group is the network model based on FCN. For example, Li et al. [10] constructed FCN with jumping connection part and introduced active learning into retinal vessel segmentation. The network model based on FCN can obtain higher-level features, but the spatial consistency of pixels is ignored in pixel segmentation. The third group is the network model based on U-Net [11]. For example, Li et al. [12] proposed IterNet, using standard U-Net as infrastructure and then discovering more details of blood vessels through iterative simplified U-Net to connect broken blood vessels. The network model based on U-Net can capture local and global information through a connection feature graph to make better decisions, so it can obtain better segmentation results. The fourth group is network architecture based on multiple models. For example, Zhang et al. [13] used M-Net [14] as the main framework to extract the structural information of vessel images and used a simple network to extract the texture information of vessel images. The multimodel network can improve performance, but it has the disadvantages of difficult training and large computation.

In recent years, more and more algorithms in the field of medical image processing focus on acquiring multiscale feature information. For example, Mu et al. [15] segmented COVID-19 lung infections by using a multiscale multilayer feature recursive aggregation (mmFRA) network. Xiao et al. [16] proposed a multiview hierarchical segmentation network for brain tumor segmentation. In this paper, we propose an improved U-Net-based fundus vessel segmentation algorithm. The main contributions of this paper are summarized as follows. (1) The improved position attention module (PA) and channel attention module (CA) were added in the jump connection part to improve the effect of vessel segmentation under low contrast. In this paper, an improved attention mechanism is added in both the encoding part and the upsampling part to improve the semantic information contained in the feature graph and improve the segmentation performance of the algorithm. (2) GCN + BR [17] was used to replace the traditional CNN to improve the ability of the algorithm to segment vascular boundaries. ConvLSTM [18] was added in the decoding part to solve the problems of gradient explosion and gradient disappearance, and depth separable convolution was used to reduce model parameters. (3) Multiscale input is used to effectively combine spatial information and semantic information of images of different sizes to solve the problem of vessel discontinuity. (4) A multiscale dense feature pyramid cascade module (MDASPP) is proposed to expand the acceptance domain. MDASPP can effectively combine feature information of feature maps with different resolutions to improve the performance of vessel segmentation through dense dilated convolution operations of different sizes.

The rest of this article is organized as follows.  Section 2 introduces the implementation principles of ConvLSTM, DenseNet, and GCN + BR in detail.  Section 3 presents the details of the proposed method.  Section 4 shows the results and performance analysis of this algorithm. Finally, the paper is summarized in Section 5.

## 2. Related Works

### 2.1. Convolution Long Short-Term Memory

Hochreiter et al. [19] proposed that LSTM is used to solve the problem that ordinary RNN cannot solve long-term dependence and may bring gradient disappearance or gradient explosion. It has been proved that LSTM can effectively solve the problem of long sequence dependency [20–22].

Traditional LSTM has a strong data processing capability. However, the traditional LSTM cannot obtain the spatial information of the image effectively because of the full connection operation in the conversion process from input to output. Shi et al. [18] proposed the ConvLSTM model to solve this problem. This model uses convolution operation instead of full connection operation to achieve input-to-end and end-to-end conversion.

### 2.2. Dense Convolution Network

In traditional U-Net, there are a series of convolution operations to learn different types of features. However, some redundant features are learned in this continuous convolution operation. Huang [23] et al. proposed DenseNet structure to alleviate this problem.

DenseNet was inspired by the residual network ResNet [24]. They are similar in that each layer's input is related to the previous layer. The main difference is that ResNet's input for each layer is only relevant to a limited number of layers ahead, whereas DenseNet's input for each layer is relevant to all layers ahead.

### 2.3. Global Convolution Network and Boundary Refinement

Global convolution network (GCN): we introduced the GCN module to simultaneously improve the localization and classification capabilities of the network in retinal vessel segmentation. The structure of GCN is shown on the left of Figure 1. Convolution with the convolution kernel *k* × *k* is replaced by the combination of convolution operations of 1 × *k* with *k* × 1 and *k* × 1 with 1 × *k*. GCN is reduced to *O*(2/*k*) parameters compared to *k* × *k* convolution. In this experiment, the value of *k* is 3 and the activation function is ReLU.

Boundary refinement (BR): it is difficult to identify the vessel boundary because the nonvessel pixels of the vessel boundary contain some vessel pixels. We introduce the BR module to improve the segmentation ability of the network at the vessel boundary. The structure of BR is shown on the right of Figure 1. We define *S*^*∗*^ as the obtained feature map: *S*^*∗*^=*S*+*R*(*S*), where *S* is the input feature map and *R*(·) is the convolution operation whose convolution kernel is *k* × *k* and whose activation function is ReLU. Add the feature map obtained by *R*(·) and the input feature map to obtain the final feature map.

## 3. Method

### 3.1. Overview

The network model proposed in this paper is based on U-Net.  Figure 2 shows the structure of the proposed algorithm. In this paper, low-resolution feature maps are obtained through average pooling of the input feature maps so that the network model can combine the feature information of feature maps with different resolutions.

GCN + BR was used to replace the traditional CNN in each layer of the coding part to improve the ability of the algorithm to separate blood vessels from the background under the condition of low contrast. The proposed MDASPP is introduced in the last layer of the coding section to further improve the connectivity of the whole segmented vessel tree. An improved attention mechanism is introduced in the jump link part to combine the feature maps of the encoding layer containing more spatial information with those of the decoding layer containing more semantic information. At the decoding layer, ConvLSTM was used to extract feature information better to alleviate the problem of gradient explosion and gradient disappearance, and deep dilated convolution was used instead of traditional convolution to expand the acceptance domain.

### 3.2. Spatial Attention Module

PA (position attention) module is added after deconvolution operation to make the feature graph, obtained by upsampling, contain more semantic information. The structure of PA is shown on (a) of Figure 3. Compared with PA [25], the convolution operation in PA is canceled. PB ∈ ℝ^(H×W)×C^ and PC ∈ ℝ^C× (H×W)^ are the characteristic graph P ∈ ℝ^H×W×C^ obtained by reshaping operation. PB and PC get characteristic graph PS ∈ ℝ^(H×W)×(H×W)^ containing rich semantic information by matrix multiplication. PF ∈ ℝ^H×W×C^ is obtained by matrix multiplication and shaping of PS and PB. The obtained PF and P are directly operated by Add and BN to obtain the final characteristic graph PE ∈ ℝ^H×W×C^.

CA (channel attention) module is added before jump connection to make the feature graph, of the corresponding encoder, contain more spatial information. The structure of CA is shown on (b) of Figure 3. Compared with CA [25], the convolution operation in CA is canceled. CB ∈ ℝ^(H×W)×C^ and CC ∈ ℝ^C× (H×W)^ are characteristic graph C ∈ ℝ^H×W×C^ obtained by reshaping operation. CB and CC get characteristic graph CS ∈ ℝ^C×C^ containing rich spatial information by matrix multiplication. CF ∈ ℝ^H×W×C^ is obtained by matrix multiplication and shaping of CS and CB. The obtained CF and C are directly operated by Add and BN to get the final characteristic graph CE ∈ ℝ^H×W×C^.

### 3.3. Multiscale Dense Feature Pyramid Module

Due to the blurring of vessel boundary and the reflection of vessel centerline in fundus image, the characteristic information of different scales can help to better extract vessels. Yang et al. [26] proposed DenseASPP by combining DenseNet and ASPP, which can generate feature information of a larger range and scale by combining the advantages of parallel and cascading convolutional layers. This paper further expands the range of features obtained through multiscale input to help elevate blood vessels. Our method is referred to as MDASPP for short. Next, we will describe the proposed MDASPP in detail.

Figure 4 shows the structure of the MDASPP. *X*_*in*_∈ℝ^H×W×C^ is an input feature graph, which is a high-level feature graph obtained from the previous coding layer. First of all, we get *X1*_in_∈ℝ^H×W×C^ by convolution and *X2*_in_∈ℝ^H/2×W/2×C^ by average pooling and convolution. Then, DenseASPP operations with gaps of 6, 7, and 8 are performed on the high-resolution *X1*_in_ to obtain *X1*_out_∈ℝ^H×W×C^. We performed DenseASPP operation with gaps of 2, 3, and 4 on low-resolution *X2*_in_ and performed upsample operation to obtain *X2*_out_∈ℝ^H/2×W/2×C^. Finally, we connect *X1*_out_ and *X2*_out_ to obtain multiscale feature information and then through convolution operation, BN, and dropout operation to obtain the feature graph *X*_out_∈ℝ^H×W×C^ containing multiscale feature information.

## 4. Results and Discussion

### 4.1. Experimental Datasets

The proposed method is tested on two common datasets of retinal fundus vessels, DRIVE [27] and CHASE_DB1 [28]. The DRIVE dataset includes 40 color fundus images of the retina, each with a size of 584 × 565. In this paper, the first 20 images of 40 images are used for training, and the other 20 images are used for testing. There are 28 retinal color images in the CHASE_DB1 dataset, each with a size of 999 × 960. In this paper, the first 14 images are used for training, and the other 14 images are used for testing.

Since increasing the amount of data in deep learning can improve the generalization ability of the model [29], this paper implements data enhancement through rotation and mirror operation on the training set. For the training set of DRIVE and CHASE_DB1, after expansion, the whole training set has 1200 images and 1680 images, respectively. Then, the data-enhanced images are sliced, and each image is cut into 64 × 64 patch blocks. Finally, the DRIVE training set is expanded into 120000 patch blocks of 64 × 64 size. The CHASE_DB1 training set is expanded into 168000 patch blocks of 64 × 64 size. In this article, 80% of it is used for training and the remaining 20% is used for verification. The test set images are only preprocessed and sliced, and no data enhancement is carried out. The patch blocks of 64 × 64 sizes obtained by the algorithm are then merged into the corresponding images.

### 4.2. Experimental Environment and Evaluation Indexes

The experiment in this paper is carried out under Keras 2.3.1. Using the binary cross-entropy loss function, the learning rate is initialized to 0.1. If the loss of the verification set remains unchanged after each epoch, the learning rate will be reduced by 10 times. The Adam optimizer is used to update the parameters; the optimal model saved in this paper takes the model with the least loss of the verification set. For DRIVE and CHASE_DB1 datasets, the Batchsize for training and testing is 8 and 16, respectively.

In this paper, sensitivity *Se*, accuracy *Ac*, F1-score, and AUC (area under the curve) are selected to evaluate the performance of the algorithm. They are defined as follows:

(1) $$\begin{array}{c} \;Se=\frac{TP}{\left(TP+FN\right)}\;,\\ Ac=\frac{\left(TP+TN\right)}{\left(TP+FN+FP+TN\right)},\\ F1-\text{Score}=\frac{2^{*}Se^{*}\left(TP/\left(TP+FP\right)\right)}{Se+\left(TP/\left(TP+FP\right)\right)}, \end{array}$$

where the True-Positive, *TP*, indicates the number of pixels that correctly classify the blood vessels and the True-Negative, *TN*, indicates the number of pixels that correctly classify the background. The False-Positive, *FP*, indicates the number of pixels that misclassify the background and the False-Negative, *FN*, indicates the number of pixels that misclassify blood vessels.

This paper is also evaluated by the Receiver-Operating-Characteristic (ROC) curve of the subjects' working characteristics. The ROC curve takes the TP as the ordinate and the FP as the Abscissa. Area-under-ROC-curve (AUC) is the area between the ROC curve and the horizontal axis, and the closer the value of AUC is to 1, the better the segmentation ability of the model.

### 4.3. Experimental Results

#### 4.3.1. Image Preprocessing

In this paper, the fundus retina image is preprocessed to improve the contrast between blood vessels and the background. The specific steps are as follows:

- The fundus retinal vascular image in the form of RGB was converted into the corresponding grayscale image.
- The grayscale image is equalized by an adaptive histogram. In this paper, the threshold of color contrast is set to 10.0, and the grid size for pixel equalization is set to (8, 8).
- The retina image is corrected by local adaptive gamma correction. In this article, the gamma factor is set to 1.0.

The preprocessing results are shown in Figure 5. It can be seen that, after preprocessing, the contrast between the blood vessel and the background is increased, and the problem of vascular centerline reflex is also suppressed.

The results of preprocessing on the dataset are shown in Table 1. It can be seen that the accuracy after pretreatment is higher than that without pretreatment, especially the sensitivity. It can be shown that through preprocessing to improve the contrast between blood vessels and background, the network can more easily learn the difference between blood vessels and background, thus reducing the number of pixels in which the background is mistakenly divided into blood vessels.

#### 4.3.2. Ablation Experiment

To verify that the improved strategy proposed in this paper can effectively improve the segmentation performance of the algorithm on retinal vessels, three groups of comparative experiments are done to show that the addition of GCN + BR, CA + PA, and MDASPP can improve the segmentation performance of the algorithm to an extent.

The results of various improvement strategies are shown in Table 2, where A1 is the result of U-Net, A2 is the result of ConvLSTM_Mnet, A3 is the result of GCN + BR + A2, A4 is the result of CA + PA + A3, and A5 is the result of MDASPP + A4. As can be seen from Table 2, the segmentation performance is improved by adding multiscale input and ConvSLTM to the traditional U-Net [10] and by adding GCN + BR, SA + PA, and MDASPP algorithms. Finally, the algorithm proposed in this paper increases the evaluation index Se, Ac, AUC, and F1-score by 7.79%, 1.68%, 1.21%, and 1.49% on the DRIVE dataset and 1.8%, 1.3%, and 7.34% on the CHASE_DB1 dataset by the evaluation index Ac, AUC, and F1-score, respectively. It is worth mentioning that the MDASPP added in this article reduces the model parameters, reduces the number of parameters by 37%, and improves the performance. The results are shown in Table 3.

#### 4.3.3. Comparison of the Results of Different Algorithms

In this paper, the proposed segmentation algorithms are compared with some most advanced algorithms on the DRIVE dataset and CHASE_DB1 dataset. The comparison results of different segmentation algorithms on the DRIVE dataset and CHASE_DB1 dataset are shown in Tables 4 and 5, respectively. The performance of the algorithm in the table is the performance in the corresponding article.

As can be seen from Table 4, the evaluation results of Se, Ac, AUC, and F1-score on the DRIVE dataset are 83.16%, 96.99%, 98.76%, and 82.91%, respectively, which are better than other algorithms. Compared with the benchmark U-Net, all indicators have achieved better performance, and there is a large gap. As can be seen from Table 5, the evaluation results of Ac, AUC, and F1-score on the CHASE_DB1 dataset are 97.51%, 99.01%, and 83.55%, respectively, which are better than other algorithms. Compared with the benchmark U-Net, three of the four metrics have achieved better performance, except that Se is lower than U-Net. To better illustrate the effectiveness of the proposed algorithm, Figure 6 shows the visual segmentation results of the proposed method on two datasets. Among them, the first list is the original RGB fundus retina image, the second column is the GT image, the third column is the segmentation result of U-Net, and the fourth column is the result of this algorithm. The first two lines show the predicted results on the DRIVE dataset, and the last two lines show the predicted results on the CHASE_DB1 dataset. It can be found that this algorithm can identify the main parts of blood vessels, and more vascular endings can be found compared with U-Net. The above results show the powerful capability of the proposed algorithm in vascular segmentation.

## 5. Conclusion

The main purpose of this paper is to improve the algorithm for fundus retinal vascular segmentation. In this paper, multiscale input and MDASPP are introduced to obtain vascular feature information of different sizes to better learn the features around vessels and improve the segmentation effect. By adding the attention mechanism to the decoding layer and the coding layer at the same time in the jump connection part, the vascular morphological information contained in the coding layer feature map and the semantic information contained in the decoding layer feature map are enhanced. In the coding part, GCN + BR is added to replace the traditional convolution to improve the ability to segment vascular boundaries. In the decoding part, ConvLSTM was added to prevent gradient disappearance and gradient explosion, and depth dilated convolution was used to enlarge the receiver domain and reduce the number of parameters. Compared with the existing advanced methods, this paper has achieved better performance.

## Figures and Tables

**Figure 1:** Global convolution network (a) and boundary refinement (b).

**Figure 2:** Network mechanism.

**Figure 3:** Attention module. (a) Position attention module (b) Channel attention module.

**Figure 4:** Multiscale DenseASPP. AVGPOOL is an average pooling operation. The rate represents the dilated rate. UPSAMPLE stands for upsampling. BN + Drop stands for batch normalization and dropout operations.

**Figure 5:** Preprocessing result.

**Figure 6:** Segmentation results of different models.

**Table 1:** Comparison of preprocessing results.

Dataset	Method	Se (%)	Ac (%)	AUC (%)	*F*1-score (%)
DRIVE	Unpreprocessing	81.78	96.99	98.74	82.67
	Preprocessing	**83.24**	**96.99**	**98.77**	**82.91**
CHASE_DB1	Unpreprocessing	80.12	97.48	99.00	83.48
	Preprocessing	**81.49**	**97.51**	**99.01**	**83.55**

The best values of Se, Ac, AUC, and *F*1-score are shown in bold.

**Table 2:** Comparison of segmentation algorithms of several improved strategies.

Method	DRIVE				CHASE_DB1			
	Se (%)	Ac (%)	AUC (%)	*F*1-score (%)	Se (%)	Ac (%)	AUC	*F*1-score (%)
A1 [22]	75.37	95.31	97.55	81.42	82.88	95.78	97.72%	77.83
A2	82.96	96.94	98.69	82.61	81.13	97.48	98.95%	82.97
A3	83.08	96.96	98.73	82.77	81.25	97.49	98.97%	83.50
A4	83.11	96.97	98.75	82.82	81.37	97.50	98.99	83.52
A5	**83.16**	**96.99**	**98.76**	**82.91**	**81.49**	**97.51**	**99.01%**	**83.55**

**Table 3:** Comparison of parameters before and after the addition of MDASPP.

Method	Number of parameters
GCN + BR_SA + PA_ConvLSTM_Mnet	14,223,095
Proposed method	**9,029,111**

The less number of parameters is shown in bold.

**Table 4:** The results of different algorithms in the DRIVE dataset.

Dataset	Methods	Year	Se (%)	Ac (%)	AUC (%)	*F*1-score (%)
DRIVE	R2U-Net [30]	2018	77.92	95.56	97.84	81.71
	U-Net [30]	2018	75.37	95.31	97.55	81.42
	LadderNet [31]	2018	78.56	95.61	97.93	82.02
	DUNet [32]	2019	78.94	96.97	98.56	N/A
	DEU-Net [33]	2019	79.40	95.67	97.72	82.70
	AG-Net [34]	2019	81.00	96.92	98.56	N/A
	IterNet [12]	2019	77.35	95.73	98.16	82.05
	BCDU-Net [35]	2019	80.07	95.60	97.89	82.24
	Tang et al. [36]	2020	81.60	95.54	97.99	N/A
	Lü et al. [37]	2020	80.62	95.47	97.39	N/A
	SA-UNet [38]	2020	82.12	96.98	98.64	82.63
	Zhang et al. [13]	2020	81.51	96.95	98.63	N/A
	RVSeg-Net [39]	2020	81.07	96.81	98.17	N/A
	Proposed method	2021	**83.16**	**96.99**	**98.76**	**82.91**

**Table 5:** The results of different algorithms in the CHASE_DB1 dataset.

Dataset	Methods	Year	Se (%)	Ac (%)	AUC (%)	*F*1-score (%)
CHASE_DB1	R2U-Net [30]	2018	77.92	95.56	97.84	81.71
	U-Net [30]	2018	**82.88**	95.78	97.72	77.83
	LadderNet [31]	2018	79.78	96.56	98.39	80.31
	DEU-Net [33]	2019	80.74	96.61	98.12	80.37
	IterNet [12]	2019	80.73	96.55	98.51	80.73
	AG-Net [34]	2019	81.86	97.43	98.63	N/A
	Lü et al. [37]	2020	81.35	96.17	97.82	N/A
	RVSeg-Net [39]	2020	80.69	97.26	98.33	N/A
	Proposed method	2021	81.49	**97.51**	**99.01**	**83.55**

The best values of Se, Ac, AUC, and *F*1-score are shown in bold.

## Data Availability

We used third-party data and therefore do not own the data. These two common datasets of retinal fundus vessels, DRIVE and CHASE_DB1, can be downloaded from the following references [27, 28].
